# Enhanced therapeutic effect of an antiangiogenesis peptide on lung cancer in vivo combined with salmonella VNP20009 carrying a Sox2 shRNA construct

**DOI:** 10.1186/s13046-016-0381-4

**Published:** 2016-07-02

**Authors:** Changhong Zhao, Junjin He, Haoran Cheng, Zhaohao Zhu, Hanmei Xu

**Affiliations:** The Engineering Research Center of Peptide Drug Discovery and Development, China Pharmaceutical University, 24 Tongjia Xiang, Nanjing, 210009 People’s Republic of China; State Key Laboratory of Natural Medicines, Ministry of Education, China Pharmaceutical University, 24 Tongjia Xiang, Nanjing, 210009 People’s Republic of China

**Keywords:** Sox2, Lung cancer, Antiangiogenesis, *Salmonella typhimurium*, Apoptosis

## Abstract

**Background:**

HM-3 is a polypeptide inhibiting angiogenesis. Recent reports suggest that the antitumor effect of angiogenesis inhibitors administered alone might be limited. Cancer stem cells can survive the lack of oxygen and nutrients. To achieve better anti-tumor effect, HM-3 was administered in combination with the attenuated *Salmonella typhimurium* VNP20009 transformed with a shRNA construct against sex determining region Y-box 2 (Sox2).

**Methods:**

Cell invasion assay and soft agar colony formation assay were used to assess the migration and growth capability of A549 cells once Sox2 was knocked down with the shRNA construct. The shRNA construct targeting Sox2 was transformed into VNP20009. After the mouse xenograft model of A549 was established, HM-3 was co-administered with VNP20009 carrying the shRNA construct. The growth of tumor was checked to compare the effectiveness of different therapies. Western blotting assay and immunohistochemistry staining of the tumor tissue were used to measure the levels of proteins associated with the apoptosis pathway.

**Results:**

Sox2 was necessary for the migration and growth of A549 cells. The expression of Sox2 was down regulated in the tumor tissue of the combined treatment group of HM-3 with VNP20009 carrying the Sox2 shRNA construct. Together with the accumulation of salmonella in tumor and the inhibition of angiogenesis by HM-3, more tumor cells went through cell apoptosis with increased expression of Bax, cleaved Caspase 3 and decreased expression of Bcl2.

**Conclusions:**

The results suggest the combination of antiangiogenesis agent HM-3 with gene therapy targeting Sox2 delivered by salmonella as a promising strategy for the treatment of lung cancer.

## Background

Lung cancer is one of the leading causes of cancer-related death throughout the world. The average 5-year survival rate of non-small cell lung carcinoma (NSCLC) which accounts for 85 % of lung cancers is only 4 %, highlighting the need for more effective treatment options [1]. HM-3 is an 18-amino acid peptide generated by the fusion of the Arg-Gly-Asp (RGD) sequence to the C-terminus of an endostatin-derived peptide. Our previous research has shown that HM-3 has no effect on the growth of tumor cells in vitro. However, HM-3 can inhibit tumor growth by inhibiting angiogenesis in vivo [2, 3]. The binding of HM-3 to integrin αvβ3 expressed on the surface of vascular endothelium cells (VECs) results in the down-regulation of MEK1 and AKT1, leading to the inhibition of the migration of VECs [4–6]. HM-3 has been approved for phase I clinical study in China (Register number: CTR20150368). Recent studies reported that the antitumor effect of angiogenesis inhibitors (AIs) administered alone might be limited implicating that additional tumor targeting drugs should be co-administered with AIs [7–9].

Tumor growth is sustained by a small number of tumor-initiating cells known as cancer stem cells (CSCs). Sox2, a gene expressed at high level in stem cells, also plays a vital role in the regenesis of lung CSCs [10–12]. It has been reported that the growth and metastasis of certain cancer cells were suppressed when Sox2 was down regulated suggesting Sox2 may be a potential target for cancer treatment [13, 14]. Finding an effective way to deliver Sox2 shRNA constructs into lung cancer cells may achieve better anti-tumor effect. Among the gene therapy delivery systems reported, attenuated salmonella offers more advantages as it can preferentially accumulate and amplify in solid tumor with little toxicity to normal organs. Also, it has been used as gene therapy delivering system for many shRNA constructs targeting different genes such as indoleamine 2, 3-dioxygenase 1 (IDO1) [15], multiple drug resistance 1 (MDR1) [16] and murine double minute 2 (MDM2) [17].

Here, we explored the antitumor effect of the novel combination therapy of HM-3 with VNP20009 carrying a Sox2 shRNA construct in a mouse xenograft model of NSCLC. Our results showed that the combined therapy had the optimal antitumor effect compared to HM-3 alone or docetaxel alone. The optimal therapeutic effect was achieved through accumulation of VNP20009 in tumor tissue, suppression of the expression of Sox2 and inhibition of angiogenesis in tumors. More tumor cells went through cell apoptosis in the combined treatment group. Also, no apparent toxic side-effect was observed in the mice.

## Methods

### Cell lines, animals and drugs

The NSCLC cell line A549 was purchased from Shanghai Institute of Cell Biology, Chinese Academy of Sciences (Shanghai, China). A549 cells were maintained in RPMI-1640 medium containing 10 % FBS. Athymic BALB/c nude female mice (5 weeks) were purchased from CAVENS (Changzhou, China). HM-3 (sequence: IVRRADRAAVPGGGGRGD) with purity of more than 99 % was chemically synthesized in our lab. The antibodies against Sox2 and CD31 were purchased from Santa Cruz (Dallas, USA). The antibodies against Bax and Bcl2 were obtained from Wanleibio (Dalian, China). The antibody against cleaved Caspase 3 was obtained from Elabscience (Wuhan, China). Docetaxel Injection was purchased from Hengrui (Jiangsu, China).

### Plasmids and bacterial strains

The mammalian shRNA expression plasmid (pGPU6/Neo) targeting Sox2 was constructed by GenePharma (Shanghai, China). The shRNA sense sequence targeting Sox2 was TGGACAGTTACGCGCACATGA as reported and the scrambled shRNA sense sequence was GTTCTCCGAACGTGTCACGT [18]. The scrambled shRNA construct was referred as shScr while the Sox2 shRNA construct was referred as shSox2. The shRNA construct was electroporated into VNP20009 with a Gene Pulser Xcell system (Bio-Rad) at 2.5 kV, 186 ohms [15]. VNP20009 transformed with the shScr (shScr-V) and VNP20009 transformed with the shSox2 (shSox2-V) was cultured in Luria-Bertani (LB) broth supplemented with ampicillin (50 μg/ml) [19]. The shRNA constructs were isolated and the targeting sequence was confirmed by sequencing. To calculate the number of colony forming unit (cfu) in culture, an optical density of 1.0 measured at 600 nm equal to 10^9^ cfu/ml was used.

### Cell invasion assay and soft agar colony formation assay

The cell invasion assay was performed using 24-transwell chambers (Corning, Newyork, USA). The procedures were carried out as previously reported [12]. For soft agar colony formation assay, a layer of media with 0.5 % agarose was first plated onto the bottom of a 6-well plate. 1 × 10^4^ cells/well were plated in a top layer of media with 0.33 % agarose. After stained with 0.005 % crystal violet, images were taken under an inverted microscope (Olympus IX53) after three weeks. The number of colonies was counted from multiple random fields.

### Tumor models and treatment

2 × 10^6^ A549 cells were injected subcutaneously (s.c) on the right flanks of the nude mice. The width (W) and length (L) of each tumor was measured with a vernier caliper. Tumor volume (TV) was determined with the formula: TV = L × W^2^/2. When the mean tumor volumes reached 300 mm^3^, the mice were randomly assigned into seven groups (*n* = 6 at least): (1) the mice received 200 μl normal saline (NS) intravenously as the normal control; (2) 2.5 × 10^6^ cfu of shScr-V diluted in NS was administered intravenously on day 1; (3) 2.5 × 10^6^ cfu of shSox2-V diluted in NS was administered intravenously on day 1; (4) HM-3 diluted in NS was administered intravenously at a dose of 3 mg/kg/day; (5) both HM-3 and shScr-V was administered as for their individual treatment regimens; (6) both HM-3 and shSox2-V was administered as for their individual treatment regimens; (7) docetaxel was administered intravenously at a dose of 10 mg/kg every four days for three injections. All the groups were listed in Table 1. Inhibition rate = [(tumor weight of control group – tumor weight of experimental group)/tumor weight of control group] × 100 %.

**Table 1:** Treatment groups

Group	Treatment
Mock	Normal saline (NS) was administered as control
shScr-V	VNP20009 carrying the scrambled shRNA construct was administered
shSox2-V	VNP20009 carrying the Sox2 shRNA construct was administered
HM-3	HM-3 was administered
HM-3 + shScr-V	Both HM-3 and shScr-V were administered
HM-3 + shSox2-V	Both HM-3 and shSox2-V were administered
Docetaxel	Docetaxel was administered

### Assay of VNP20009 in tissues and blood

After the A549 tumor model in nude mice was established, VNP20009 was administered by intravenous injection at a dose of 2.5 × 10^6^ cfu per mouse. On days 2, 7 and 14 after injection, tumors and major organs were aseptically removed, weighted and homogenized in PBS. 1 ml homogenized tissue of the same weight (100 mg) was diluted in gradient and 100 μl was plated onto LB agar plates containing ampicillin (50 μg/ml). In the case of blood analysis from mice, 200 μl blood was collected as the mice were killed and was plated directly onto the LB plates. The LB plates were incubated at 37 Celsius overnight and the bacteria colonies were quantified.

### Western blotting assay (WB)

The tumor samples were snapped into small pieces and incubated with RIPA cell lysis buffer supplemented with protease inhibitors on ice for 20 min. After that, the samples were homogenized with a glass tissue grinder. After centrifuging (14,000 × g) for 20 min, the supernatant was removed and boiled with protein loading buffer. The western blotting was carried out as described before [5]. ImageJ software (Wayne Rasband, USA) was used to analyze the result. The relative protein expression was calculated by dividing the optical density of the protein analysed with the optical density of β-actin of the same group. The results of three independent experiments were calculated.

### Immunohistochemistry (IHC)

Tumor and organ tissue was fixed in 4 % formalin and embedded in paraffin. Sections were deparaffinized and rehydrated. For hematoxylin and eosin (H&E) staining, sections were stained in hematoxylin and then counterstained with eosin. For immunohistochemistry staining, after treatment with 3 % H_2_O_2_, sections were boiled in 10 mM sodium citrate buffer (pH 6.0) for antigen retrieval. After blocking, sections were incubated with the primary antibody as recommended by the supplier, washed with PBS, and then incubated with the horseradish peroxidase labeled secondary antibody. Sections were finally incubated with DAB and counterstained with hematoxylin.

### Statistical analysis

All the data was collected and processed with the Statistical Program for Social Sciences (SPSS version 13.0, Chicago, USA). The difference between samples of the same group was tested by one-way analysis of variance. It would be considered statistically significant when *P* < 0.05 and statistically highly significant when *P* < 0.01.

## Results

### The invasion and anchorage-independent growth capability of A549 cells was inhibited as Sox2 was knocked down

To confirm the effectiveness of the shRNA constructs, the expression of Sox2 at protein level in A549 cells was analysed with WB after transfected with the shRNA constructs. Compared to the A549 cells transfected with shScr, the expression of Sox2 was reduced by more than 80 % in the cells transfected with shSox2 (Fig. 1a, *P* < 0.01). The number of cells that migrated was 236.33 ± 26.08 for A549 cells transfected with shScr, while it was 45.23 ± 12.50 for A549 cells transfected with shSox2 (Fig. 1b, *P* < 0.01). The number of colonies that formed was 225.33 ± 62.98 for A549 cells transfected with shScr, while it was 57.33 ± 12.01 for cells transfected with shSox2 (Fig. 1c, *P* < 0.05). Sox2 plays an important role in regulating the migration and anchorage-independent growth of A549 cells. Therefore, Sox2 may be considered as a potential target for the treatment of lung cancer.

**Fig. 1:** The migration and proliferation potential of A549 cells was inhibited as Sox2 was down regulated. **a** The expression of Sox2 at protein level in A549 cells was analysed using western blot after transfection. shScr, A549 cells transfected with shScr. shSox2, A549 cells transfected with shSox2. The quantification assay of WB results was shown as mean ± SD obtained from three repeated experiments. ** *P* < 0.01 vs shScr group. **b** The migration capability of A549 cells was reduced after transfected with shSox2. Original magnification × 200. The quantification data shown was mean ± SD obtained from three fields. ** *P* < 0.01 vs shScr group. **c** The colony forming capability of A549 cells was inhibited after transfected with shSox2. Original magnification × 200. The quantification data shown was mean ± SD obtained from three fields. * *P* < 0.05 vs shScr group

### VNP20009 selectively accumulated in tumors

To ensure that VNP20009 transformed with the shRNA expression plasmid still preferentially accumulated in solid tumor tissues, the distribution of shScr-V in the A549 xenografts and major organs of mice treated with shScr-V was monitored. On days 2 post-injection, the amount of shScr-V in tumors was significantly higher than it was in spleen and other organs (Fig. 2a). No shScr-V was detected in the blood on days 2 suggesting that the environment in blood was not well adapted by VNP20009 [20]. Quantitative analyses showed that on days 2, 7 and 14 after injection, shScr-V could maintain its accumulation in tumors over spleen and other organs at a ratio greater than 1000:1 (Fig. 2b, *P* < 0.01).

**Fig. 2:** VNP20009 preferably accumulated in tumors in vivo. **a** The representative images of LB agar plates planted with different homogenized tissue after serial dilution or blood on days 2 after injection. The dilution factor was marked, 1/10 for ten fold dilution. **b** The quantitative analyses of the bacterium count by cfu/g tissue were presented for days 2, 7 and 14 post injections. Data shown was mean ± SD obtained from three independent experiments. * *P* < 0.01 vs the tumor group on days 2, Δ*P* < 0.01 vs the tumor group on days 7, #*P* < 0.01 vs the tumor group on days 14

### Antitumor activity of HM-3 combined with shSox2-V in vivo

After the mouse xenograft model of A549 was established, the mice were assigned randomly to seven groups (Fig. 3a and Table 1). HM-3 was administered alone and in combination with shScr-V or shSox2-V. Although the tumor growth of the shSox2-V, HM-3 + shScr-V and docetaxel groups all had been suppressed compared to the mock group (*P* < 0.05, respectively), the best therapeutic effect was obtained in the HM-3 + shSox2-V group (Fig. 3b, *P* < 0.01). The mean tumor volume of the HM-3 + shSox2-V group was 682.37 mm^3^, while that in the mock, shScr-V, shSox2-V, HM-3, HM-3 + shScr-V and docetaxel groups was 1516.32 mm^3^, 1194.84 mm^3^, 1043.85 mm^3^, 1129.68 mm^3^, 906.14 mm^3^ and 822.78 mm^3^ respectively at the end of the treatment (Fig. 3c). The difference of tumor volume between the HM-3 + shScr-V and HM-3 + shSox2-V group was statistically significant (*P* < 0.05) implicating that the shSox2 carried by shSox2-V contributing to the inhibition of tumor growth. The mean weight of tumors of the HM-3 + shSox2-V group was 0.586 g, while that in the mock, shScr-V, shSox2-V, HM-3, HM-3 + shScr-V and docetaxel groups was 1.420 g, 1.075 g, 0.899 g, 1.037 g, 0.783 g and 0.737 g respectively (Fig. 3d). Both shScr-V and shSox2-V could enhance the antitumor effect of HM-3 as compared to the mock group (*P* < 0.05 and *P* < 0.01, respectively). The best antitumor effect was achieved in the HM-3 + shSox2-V group. Due to the variance of tumor weight in mice, the difference of tumor weight between the HM-3 + shScr-V and HM-3 + shSox2-V group was not statistically significant.

**Fig. 3:** Inhibition of A549 tumor growth by various treatments in vivo. **a** Images of the tumor-bearing mice of each group. **b** Images of the tumors of each group at the end of treatments. **c** The mean tumor volume of each group over the 18-day treatment period. **d** Tumor wet weights of each group were measured after the animals were killed. Data was shown as mean ± SD obtained from each group. * *P* < 0.05 vs Mock group, ** *P* < 0.01 vs Mock group, Δ*P* < 0.05 vs HM-3 + shScr-V group

### The expression of Sox2 and microvessel formation in the A549 xenografts of different treatment groups

The expression of Sox2 in the tumor tissues was examined by WB and IHC. In contrast to the groups treated with NS, HM-3 and shScr-V, Sox2 expression was much lower in the HM-3 + shScr-V, HM-3 + shSox2-V and docetaxel groups (Fig. 4a, *P* < 0.05). When co-administered with HM-3, shSox2-V could more effectively inhibit the expression of Sox2 compared to shScr-V (*P* < 0.01). The results indicated that the successful transfection of Sox2 shRNA by VNP20009 in vivo. Docetaxel is a microtubule inhibitor that inhibits the disassociation of microtubule during cell division. The down regulation of Sox2 in the docetaxel group might result from the cell cycle arrest and cell death induced by docetaxel rather than a direct effect. In consistent with the WB result, the number of Sox2 positive cells was also reduced in the HM-3 + shScr-V, HM-3 + shSox2-V and docetaxel groups (Fig. 4b). The number of Sox2 positive cells per field for the mock, shScr-V, shSox2-V, HM-3, HM-3 + shScr-V, HM-3 + shSox2-V and docetaxel groups was 39.5, 39.25, 30.75, 41.75, 22.25, 10.5 and 13.25 respectively (Fig. 5a).

**Fig. 4:** Expression of Sox2 and CD31 in the tumors of each treatment group. **a** The expression of Sox2 and CD31 were examined with WB assays. The quantification assay of WB results was also presented. Data shown was mean ± SD obtained from three independent experiments. * *P* < 0.05 vs Mock group, #*P* < 0.01 vs HM-3 + shScr-V group. **b** The representative images of IHC staining for Sox2 of tumors treated in each group. **c** The representative images of IHC staining for CD31 of tumors treated in each group

**Fig. 5:** The quantification analysis of the IHC result. **a** The Sox2 positive cells per field were counted. The data shown was mean ± SD obtained from four fields. * *P* < 0.05 vs Mock group, Δ*P* = 0.055 vs HM-3 + shScr-V group. **b** The microvessel number per field was counted. The data shown was mean ± SD obtained from four fields. * *P* < 0.05 vs Mock group

CD31 has been used extensively to evaluate the degree of angiogenesis in tumors. As shown in the WB and IHC results, the amount of CD31 was much lower in the HM-3, HM-3 + shScr-V and HM-3 + shSox2-V groups compared to those treated with NS, shScr-V, shSox2-V and docetaxel (Fig. 4a and c, *P* < 0.05). The microvessel number per field for the mock, shScr-V, shSox2-V, HM-3, HM-3 + shScr-V, HM-3 + shSox2-V and docetaxel groups was 10.25, 9.75, 10.75, 3.5, 3.25, 2.5 and 9.75 respectively (Fig. 5b). The results confirmed that HM-3 could inhibit the microvessel formation in tumors. The difference of microvessel density between HM-3 + shScr-V and HM-3 + shSox2-V group was not significant suggesting that the antiangiogenesis activity of HM-3 was not affected in both groups.

### Effects of HM-3 with shSox2-V on the expression of apoptosis-related protein in the A549 xenografts

Histological examination showed large areas of necrosis in the HM-3 + shScr-V, HM-3 + shSox2-V and docetaxel groups (Fig. 6a). The accumulation of salmonella and co-expression of Sox2 shRNA enhanced the therapeutic effect of HM-3 on the growth of tumor. It has been reported that the silencing of Sox2 leading to the up regulation of apoptotic marker cleaved Caspase 3 (C-caspase 3) in lung cancer [21]. Also, it has been found that VNP20009 could migrate away from vasculature and induce apoptosis in tumor tissue [22]. Together with HM-3 inhibiting the microvessel formation in tumors, we assumed that tumor cells were more susceptible to the induction of cell death. The expression of apoptosis-related protein C-caspase 3, Bax and Bcl2 was examined with WB (Fig. 6b). Compared to the mock group, the expression of apoptosis stimulators Bax and C-caspase 3 was much higher in the HM-3 + shSox2-V and docetaxel groups (*P* < 0.05). In contrast, the expression of apoptosis inhibitor Bcl2 was much lower in the HM-3 + shSox2-V and docetaxel groups (*P* < 0.05). Those results suggested that the apoptosis pathway was activated in the HM-3 + shSox2-V and docetaxel groups. The difference of the expression of Bax and C-caspase 3 between the HM-3 + shScr-V and HM-3 + shSox2-V group was statistically highly significant (*P* < 0.01, respectively) indicating that shSox2 contributed to the activation of the apoptosis pathway.

**Fig. 6:** The induction of cell apoptosis in tumors. **a** Representative images of H&E staining of tumors of each treatment group. **b** The expression of Bax, Bcl2 and cleaved Caspase 3 (C-caspase 3) were examined with WB assays. The quantification assay of WB results was also presented. The data shown was mean ± SD obtained from three independent experiments. * *P* < 0.05 vs Mock group, #*P* < 0.01 vs HM-3 + shScr-V group

### Systematic toxicity in the mice treated with HM-3 + shSox2-V

Previous study has found that VNP20009 administered alone can be tolerated by athymic mice [23]. The systematic safety when HM-3 and shSox2-V administered together still requires further verification. We compared the body weight of mice in the HM-3 + shSox2-V group to the other groups (Fig. 7a). Those mice treated with docetaxel had the lowest mean body weight at the end of the study. The body weight of the mice treated with HM-3 was about the same as the mock group. Although the mean body weight of mice in the HM-3 + shSox2-V group was lower than the mock group, the difference was not statistically significant. After the tumor-bearing mice were sacrificed, their hearts, livers, spleens, kidneys and lungs were harvested and examined by H&E staining (Fig. 7b). As shown in the result, the combined treatment with HM-3 and shSox2-V had little toxicity to the major organs compared to the mock group.

**Fig. 7:** Systematic toxicity in the mice of each treatment group. **a** The mean body weight of tumor-bearing mice treated in each group was measured during the study. The data shown was mean ± SD obtained from each group. **b** The images of H&E staining of major organs of mice treated with NS and HM-3 + shSox2-V

## Discussion

At the early stages of tumor progression, microvessels are formed around tumor. If angiogenesis inhibitors are administered at this stage, the growth of tumor could be effectively inhibited. However, the microenvironment in the inner tumor mass changes as tumor progresses. The actions of antitumor drugs may be affected as the expression of various factors and microRNAs are influenced by the microenvironment [24, 25]. Also, the survival of CSCs further limits the effectiveness of chemotherapy and anti-angiogenesis therapy [26–28]. In this study, the treatment was started after the tumor volume was greater than 300 mm^3^. On one hand, polypeptide HM-3 was administered to suppress the microvessel formation in tumor which cut the supply of oxygen and nutrients for tumor growth. On the other hand, attenuated facultative anaerobe VNP20009 was administered which can specifically accumulate in tumor because of its natural tropism for hypoxic areas in contrast to chemo drugs [29]. The inhibition of microvessel formation in tumor could not affect the tumor targeting potential of VNP20009 as it was cleared away from the blood quickly and accumulated in tumors shortly after injection. To further inhibit the survival of CSCs in tumor tissue, a shRNA construct targeting Sox2 was transformed into VNP20009. The expression of Sox2 was down regulated in the tumor tissue of the combined treatment group while with much smaller tumor volume.

The engineered salmonella enhanced the antitumor effect of HM-3 on lung cancer compared to the individual therapy group. The inhibition rate of the HM-3 + shSox2-V group was 58.73 %, while that in the shScr-V, shSox2-V, HM-3, HM-3 + shScr-V and docetaxel groups was 24.3 %, 36.69 %, 26.97 %, 44.86 % and 48.1 % respectively. Our results suggested that this combination was effective in inhibiting tumor growth in vivo. According to our knowledge, this was the first report that attenuated salmonella with a shRNA construct targeting Sox2 was co-administered with a polypeptide inhibiting angiogenesis in the treatment of lung cancer.

Sox2 is a poor prognostic indicator in stage I lung cancer [30]. Also, it has been reported that the expression of Sox2 promoted drug resistance of certain tumors [31, 32]. By knocking down the expression of Sox2 with shRNA, the growth of lung cancer cells was inhibited. In consistent with previous reports, the down regulation of Sox2 was related to the expression of apoptosis related marker C-caspase 3 [21]. However, our results suggested that knocking down Sox2 alone was not enough to significantly inhibit A549 tumor growth in vivo. Considering the redundancy of signaling factors in tumor cells, other members of the same protein family or different pathways may compensate for the loss of Sox2 leading to the survival of tumor cells [33, 34].

Cell death mediated by apoptosis is important in the regulation of tumor growth. It has been reported that VNP20009 could migrate from the vascular and induce apoptosis in tumor [22]. Our results showed that the apoptosis induced by VNP20009 alone was not evident. This might be due to the difference of tumor model and treatment regimens. More tumor cell went through apoptosis in the HM-3 + shSox2-V group implicating that the inhibition of angiogenesis by HM-3 had synergistic antitumor effects with shSox2-V. The cell apoptosis pathway was also activated in the group treated with docetaxel due to its cytotoxicity. It has been reported that the combination therapy of cytotoxic agents with salmonella was effective in inhibiting the growth of prostate cancer [17]. However, whether this combination can be applied to lung cancer still requires further verification.

## Conclusions

Our study suggested that HM-3 together with a gene therapy targeting Sox2 delivered by VNP20009 was an attractive treatment option for patients with lung cancer. However, to achieve better antitumor effect, multi-targeting therapies with cytotoxic drugs and the use of other gene therapy delivering system may be considered [35]. Also, the key factors of other signal pathways that are involved in lung cancer growth can be evaluated as potential targets [36].

## Abbreviations

AIs, angiogenesis inhibitors; C-caspase 3, cleaved Caspase 3; Cfu, colony forming unit; CSCs, cancer stem cells; H&E, hematoxylin and eosin; IDO1, indoleamine 2, 3-dioxygenase 1; IHC, immunohistochemistry; L, length; LB, Luria-Bertani; MDM2, murine double minute 2; MDR1, multiple drug resistance 1; NS, normal saline; NSCLC, non-small cell lung carcinoma; RGD, Arg-Gly-Asp; s.c, subcutaneously; shScr, the scrambled shRNA construct; shScr-V, VNP20009 transformed with the shScr; shSox2, the Sox2 shRNA construct; shSox2-V, VNP20009 transformed with the shSox2; Sox2, sex determining region Y-box 2; TV, tumor volume; VECs, vascular endothelium cells; W, width; WB, western blotting assay
